# Protective Effect of Salvianolic Acid A against N-Methyl-N-Nitrosourea-Induced Retinal Degeneration

**DOI:** 10.1155/2022/1219789

**Published:** 2022-05-27

**Authors:** Yumei Zhou, Weiwei Xu, Anqi Liu, Ye Tao, Qun Wang, Yanfeng Yang, Liqiang Wang, Yifei Huang

**Affiliations:** ^1^Department of Ophthalmology, Chinese PLA General Hospital, Beijing, China; ^2^Department of Ophthalmology, China Emergency General Hospital, Beijing, China

## Abstract

**Objective:**

Retinal degeneration (RD) is a serious, irreversible, and blinding eye disease, which seriously affects the visual function and quality of life of patients. At present, there is no effective method to treat RD. The final outcome of its development is photoreceptor cell oxidation and apoptosis. Therefore, looking for safe, convenient, and effective antioxidant therapy is still the key research field of Rd. In this study, the mice model of RD was induced by N-methyl-N-nitrosourea (MNU) *in vivo* to explore the therapeutic effect and mechanism of salvianolic acids (Sal A) on RD. *In vitro*, the protective effect of Sal A on MNU injured 661 W cell line of mouse retina photoreceptor cone cells was investigated preliminarily.

**Methods:**

Male C57BL/6 mice (7–8 weeks old) received a single intraperitoneal injection (ip) of 60 mg/kg MNU or vehicle control. Treatment groups then received Sal-A 0.5 mg/kg and 1.0 mg/kg via daily intravenous injections. On day 7, functional and morphological examinations were performed, including photopic and scotopic electroretinography (ERG) and hematological analyses to observe functional changes and damage to the outer nuclear layer (ONL). On the 3rd and 7th days, the levels of superoxide dismutase (SOD) activity and malondialdehyde (MDA) content were determined. The expression of retinal Bax, Bcl-2, and caspase-3 was quantified by Western blot and RT-PCR assays. 661 W strain of mice retinal photoreceptor cone cells were cultured *in vitro* and treated with 1 µm MNU. The cells in the treatment group were given 50 *μ*M Sal A as an intervention. The growth of 661 W cells was observed and recorded under an inverted light microscope, and the activity of cells was detected by the MTT method.

**Results:**

Sal A treatment was effective against MNU-induced RD in mice at both 0.5 mg/kg/d and 1.0 mg/kg/d doses, and the protective effect was dose-dependent. Sal A can alleviate MNU-mediated alterations to retinal ERG activity and can support maintenance of the thickness of the ONL layer. Sal A treatment increases the expression of retinal SOD and reduces the lipid peroxidation product MDA, suggesting that its protective effect is related to the oxidation resistance. It can offset changes to the expression of apoptotic factors in the retina caused by MNU treatment. Sal A mitigates MNU-mediated damage to cultured mice photoreceptor cone cells 661 W *in vitro*.

**Conclusion:**

Sal A alleviates the damage caused by MNU to retinal photoreceptor cells *in vivo* and *in vivo*, and its protective effect is related to its antioxidant and antiapoptotic activities.

## 1. Introduction

Retinal degeneration (RD) is a common ophthalmic condition that impairs the visual function significantly. It is characterized by progressive apoptosis, which finally results in the death of photoreceptor cells and blindness [1, 2]. Reactive oxygen species (ROS) has been considered as the key factor of photoreceptor cell apoptosis in RD [3]. ROS can activate the poly-ADP ribose polymerase (PARP) in photoreceptor nucleus, so as to regulate the expression level of apoptosis inducing factor (AIF), and finally touch the apoptosis of photoreceptor cells [4].

There is currently no effective treatment for RD yet. In recent years, a variety of *in vivo*, *in vitro*, and clinical experimental treatment methods have been studied for RD, such as traditional neurotrophic therapy, calcium antagonistic therapy, antiapoptosis/antioxidant therapy, growth factor therapy, as well as new gene therapy, stem cell therapy, retinal transplantation, artificial retina etc., which have made progress to a certain extent. However, the toxic and side effects of treatment or complex administration methods are the difficulties that limit the research of RD treatment [5–11]. So, the search for safe, convenient, and effective antioxidant therapies is an important research strategy with regard to RD. One effective means to study RD is to use chemical agents, such as N-methyl-N-nitrosourea (MNU), to make animal models. MNU is a nitrophthalamine alkylate with strong mutagenic ability that has been shown to be particularly effective in a variety of tissues [12–14]. In the field of ophthalmology, MNU has been successfully used to induce cataracts, corneal diseases, and animal models of RD [15, 16]. With regard to RD in particular, MNU has been shown to selectively induce photoreceptor cell degradation through the induction of oxidative stress *in vitro* and *in vivo* [4, 17].

In this study, we investigate the potential of salvianolic acid A (Sal A) to inhibit MNU-induced retinal photoreceptor cell apoptosis. Sal A (Figure 1) has a convenient preparation, and it is known to exert few adverse reactions *in vivo*. Because Sal A has a strong antioxidant capacity [18, 19], we predicted that it would protect the retina from damage and thus delay the occurrence and development of RD.

## 2. Materials and Methods

### 2.1. Animals

Male 7-week-old C57BL/6 mice were bought from Viton Lever Company in Beijing, China. They were kept in an air-conditioned facility with a room temperature of 18°C–23°C, humidity of 40%–65%, and a 12-hour light/dark cycle. They were fed normal chow and water ad libitum. The animal study protocol no. is 20161111.

Animal ethics statement: Our animal study was performed the ARVO's Statement on the Use of Animals in Ophthalmology and Vision Research.

### 2.2. Drugs and Reagents

MNU (Sigma; St. Louis, MO, USA) was kept at −20°C in the dark, diluted in normal saline containing 0.05 percent acetic acid, and given to mice intraperitoneally (ip) in a single dosage of 60 mg/kg. Sal A-lyophilized powder (purity >98%) was dissolved in normal saline (NS) and injected intravenously into the tails of mice.

### 2.3. Experimental Methods

#### 2.3.1. Animal Treatments

Mice were randomly divided into 5 groups (10 mice in each group). Two groups were considered control groups, and they received a single dose of vehicle (NS containing 0.05% acetic acid) ip. Mice in one of the negative control groups (NC) received a tail vein injection of NS on days 1 through 7. Mice in the other negative control group (NC + Sal-A) were injected with Sal A at a dose of 1.0 mg/kg body weight (bw) via the tail vein on each of days 1 through 7.

Mice in three of the groups received a single dose of 60 mg MNU/kg bw ip and then were treated as follows. One group of mice (the MNU group) received a tail vein injection of NS (5 mL/kg/d) on days 1 through 7. A second group of mice (the MNU + Sal A (0.5) group) received an initial injection of Sal A at a dose of 0.5 mg/kg bw into the tail vein within 1 h of MNU treatment. Then, from days 1 through 7, the mice were injected with Sal A (0.5 mg/kg bw) everyday through the tail vein. The third group of mice (the MNU + Sal A (1.0) group) were treated similarly to the MNU + Sal A (0.5) group, except that the dose of Sal A was 1.0 mg/kg bw every day.

#### 2.3.2. Electroretinogram (ERG) Analysis

After 7 days of MNU administration, the mice were examined by ERG. After 24 hr of dark adaptation, mice were anesthetized by ip injection of chlorpromazine (15 mg/kg) and ketamine 60 mg/kg (Pfizer, USA). Compound tropicamide eye drops (Santen Pharmaceuticals, Japan) were administered to dilate the pupils, and the corneas were anesthetized with cocaine hydrochloride eye drops (Santen Pharmaceutical Co., Japan). On the recording stage under dim red light, the recording electrode was placed on the limbus, and the reference electrode and the ground electrode were placed on the cheek and tail, respectively. The b-wave amplitude and latency were recorded with a single flash stimulation.

#### 2.3.3. Collection of Mice Eyeballs

After the mice were deeply anesthetized, right eyeballs were taken and fixed in 4% paraformaldehyde for 12 hours, marked at the top with toluidine blue, and then embedded in paraffin. The left eyeball was removed and preserved in liquid nitrogen.

#### 2.3.4. Histopathological Assessment of Retinal Morphology

Routine paraffin-embedded specimens were sagittally sectioned through the optic nerve, and 5 *µ*m thick sections were made. After staining with hematoxylin and eosin (HE), light microscopy (OLMPUS BX51) was used to observe the tissues, and images were analyzed with ImageView software. The thickness of the outer nuclear layer (ONL) of the retina was measured at an interval of 200 *μ*m up and down the vertical axis. Each measurement was performed 5 times.

#### 2.3.5. Determination of the Superoxide Dismutase Activity (SOD) and Malonaldehyde (MDA) Content

The retinal tissue was homogenized and centrifuged at 500 *g* for 5 minutes at 4°C in PBS containing 0.5 percent Triton X-100 (pH 7.4). The activity of superoxide dismutase (SOD) in the supernatant was determined using a SOD Assay Kit (Biyuntian Biotechnology Co., Ltd., China). The SOD activity was determined using a spectrophotometer to measure the absorbance at 560 nm, and the findings were reported in units per mg protein.

The malondialdehyde (MDA) level was determined using a colorimetric thiobarbituric acid test kit (Biyuntian Biotechnology Co., Ltd., China). The MDA intensity was determined at 532 nm using a spectrophotometer, and the lipid peroxide levels in the presence of MDA were expressed as nmol/mg protein.

#### 2.3.6. Determination of the Expression Levels of Apoptosis-Related Genes by Western Blotting and Reverse Transcription Polymerase Chain Reaction (RT-PCR) Assays

*Western Blotting.* Slices of retinal tissues were added to cell lysis solution to remove cellular proteins, which were then separated using SDS-PAGE. The transfer of the proteins to nitrocellulose membranes was prevented using 5% nonfat milk powder. Anti-Bax, anti-BCL-2, anti-caspase-3, and anti-actin primary monoclonal mouse antibodies were bought from Abcam and utilized at dilutions of 1 : 1000. The secondary antibody, goat anti-mouse IgG, was obtained and utilized at a dilution of 1 : 1000 from Biyuntian Biotechnology Co., Ltd. Photographs were taken using the gel imaging equipment, and the gray value was analyzed using the program Image J. The expression level was estimated as the ratio of the target protein's optical density to that of actin.

*RT-PCR.* The Trizol reagent was used to extract RNA from retinal tissues. Spectroscopic analysis was conducted to quantify the RNA, which was subsequently reverse-transcribed into a single-stranded cDNA. The relative expression levels of actin, Bax, Bcl-2, and caspase-3 genes were adjusted and measured using gene-specific primers and 25 cycles of cDNA amplification. The primers of Bax, Bcl-2, and caspase-3 were referenced [20].

#### 2.3.7. Cell Experiments

*Cell Grouping.* 661 W cells (from ATCC) are a mice retinal photoreceptor cone cell line. Treatments were initiated when cells reached 70% to 80% confluence. The medium was removed and replaced with fresh media-containing treatments according to 4 treatment groups, as follows. A culture medium containing 1 *µ*M MNU was added to cells of the MNU group. A culture medium containing 1 *μ*M MNU and 50 *μ*M Sal A was added to cells of the MNU + Sal-A group . A culture medium lacking additives was added to the NC (the normal control) . A culture medium containing 50 *μ*M Sal A was added to cells of the NC + Sal-A group

*Cell Growth.* Cell growth was monitored and recorded consistently with an inverted optical microscope.

*Cell Viability Assay.* The MTT method was used to find out how healthy the cells that had been treated were, and the absorbance (A) value was found by setting a spectrophotometer to 490 nm. To figure out how many cells were alive, we used this formula: cell viability (percentage) = A for treatment groups/A for control groups ×100. The average of five tests that were done again is used to figure out the result.

#### 2.3.8. Statistical Analysis

Data are expressed as mean ± standard deviation and were subjected to analysis of variance (ANOVA). Differences for which *P* < 0.05 were considered statistically significant.

## 3. Results

### 3.1. Changes to the Retinal ERG Activity

On day 7, the MNU-treated group's b-wave amplitudes of retinal ERGs were substantially lower than those of the equivalent NC group in both photopic and scotopic circumstances (*P* < 0.01, Figure 2). The b-waves of mice in the MNU group were low and flat, suggesting that MNU caused significant damage to the retinas. In the treatment groups, Sal A was found to significantly inhibit the MNU-invoked decrease of the b-wave amplitude (*P* < 0.01) in a dose-dependent manner (*P* < 0.01). The b-wave amplitude of the NC + Sal-A group was not significantly different from that of the normal control NC group, indicating that the administration of Sal A alone did not affect the electrical activity of the normal mouse retina.

### 3.2. Detection of ONL Thickness in Each Group on Day 7

The retinal ONL of the MNU-treated mice became thinner over time (*P* < 0.01, Figure 3), and the ONL layer in this group was basically eliminated by day 7. The thickness of the two Sal A treatment groups was significantly greater than that of the MNU group (*P* < 0.01), and the average ONL thickness of the MNU + Sal A (1.0) group was significantly greater than that of the MNU + Sal A (0.5) group (*P* < 0.01). There was no significant difference in the ONL layer thickness between the NC + Sal-A group and the NC group.

### 3.3. Effects of Sal A on the SOD Activity and MDA Content in Retinal Tissues

As seen in Figure 4, in the MNU-treated group, the SOD activity was considerably lowered (*P* < 0.01) and MDA content was significantly elevated (*P* < 0.01)compared to those in the NC group on day 3. The SOD activity in the retinas of both Sal A treatment groups was probably greater than that in the MNU group (*P* < 0.01), and the high-dose group had considerably increased SOD activity than the low-dose group (*P* < 0.01). MDA concentrations in the retinas of Sal A-treated mice were considerably lower than those in the MNU group (*P* < 0.01), and the high-dose group had significantly lower MDA concentrations than the low-dose group (*P* < 0.01).

On day 7 of the treatment program, the mean retinal SOD activity of the MNU group continued to decrease with time (*P* < 0.01), and the MDA level continued to increase (*P* < 0.01). While the retinal SOD activity of the two Sal A treatment groups continued to decrease (*P* < 0.01), the SOD activity in the retinas of mice treated with Sal A remained significantly higher than that of the MNU group (*P* < 0.01). MDA levels in the retinas from both treatment groups continued to increase (*P* < 0.01) but remained significantly lower than those in the MNU group (*P* < 0.01). No significant differences were found between levels of SOD or MDA in the NC groups treated with Sal A and with vehicle control (*P* > 0.05).

### 3.4. Effect of Sal A on the Expression Levels of Apoptosis-Related Genes

As illustrated in Figures 5 and 6, both Western blotting and quantitative real-time PCR experiments revealed that on day 3 of the treatment regimen, the levels of expression of the retinal proapoptotic genes Bax and caspase 3 were significantly higher in the MNU-treated group than in the NC group (*P* < 0.01). They were all considerably lower than the MNU group (*P* < 0.01), while being significantly higher than the NC group (*P* < 0.01). The expression of these genes was significantly greater in the MNU + Sal A (0.5) group than in the MNU + Sal A (1.0) group (*P* < 0.01), showing that proapoptotic genes were expressed more in the low-dose group than in the high-dose group. The antiapoptotic gene Bcl-2 expression was substantially decreased in mice treated with MNU (*P* < 0.01) compared to animals treated with NC. The Bcl-2 gene expression was considerably greater in the treatment group that received Sal A alone than in the MNU group (*P* < 0.01). The expression of this antiapoptotic gene was significantly lower in the MNU + Sal A (0.5) group than in the MNU + Sal A (1.0) group (*P* < 0.01), indicating that it was expressed less in the low-dose group than in the high-dose group. Between the NC + Sal A and NC groups, there were no significant changes in the expression of the three apoptosis-related genes (*P* > 0.05).

At day 7, the expression levels of Bax, caspase-3, and Bcl-2 were restored to normal in the MNU group, and there was no significant difference between the MNU group and the normal NC group (*P* > 0.05). On the seventh day, the ONL of the retina was essentially atrophic, and photoreceptor cells had undergone apoptosis. As a result, the observed amount of apoptotic gene expression was the same as the expression of other normal retinal structures, which was normal. While Bax and caspase 3 expression levels were considerably higher in the Sal A treatment group than in the normal control NC group (*P* < 0.01), And The two genes were expressed at a greater level in the MNU + Sal A (0.5) group than in the high-dose MNU + Sal A (1.0) group (*P* < 0.01). Both treatment groups had a lower Bcl-2 expression than the NC group (*P* < 0.01), and the MNU + Sal A (0.5) group had a lower Bcl-2 expression than the MNU + Sal A (1.0) group (*P* < 0.01). Between the NC + Sal A and NC groups, there was no significant change in the expression of the three apoptotic genes (*P* > 0.05).

### 3.5. Morphological Changes of 661 W Cells

Cells were treated in the noted ways and then were incubated for 12 hr and 24 hr after treatment, and the morphologies were then observed under light microscopy (Figure 7(a)). The adherent growth of cells in the NC group and the NC + Sal-A group was consistent with each other, and the cells were completely confluent at 24 h. On the other hand, the cells treated with MNU shrank and began to fall off at 12 h, and most cells detached from the substrate by 24 h post-treatment. In the MNU + Sal-A group, however, while a small number of cells detached from the substrate at 12 h, some cells remained adhered to the plate and grew well at 24 h.

### 3.6. Effects of Treatments on Cell Viability

The viability of cells in the MNU group, as measured by MTT assays, was significantly lower than that in the NC group at 12 h (*P* < 0.01, Figure 7(b)), and continued to decrease at 24 h (*P* < 0.01). Although the viability of cells in the MNU + Sal-A group was continued to decrease with time (*P* < 0.01), but significantly higher than cells treated only with MNU (*P* < 0.01). The viability of cells treated only with Sal A group was not significantly different from that of the NC group (*P* > 0.05), indicating that Sal A itself did not affect cell activity.

## 4. Discussion

Sal A, a water-soluble phenolic acid extracted from *Salvia miltiorrhiza*, has been demonstrated to exhibit a broad spectrum of pharmacological effects, including antioxidant and anti-inflammatory properties, myocardial ischemia protective, antithrombotic, neuroprotective, and antifibrotic effects [21–26]. In fact, Sal A has one of the strongest antioxidative effects that has been identified among natural products to date, and it has been shown to remove superoxide anions and hydroxyl radicals from the environment and to prevent lipid peroxidation [27, 28]. A study of effects of Sal A application to the eye found that it was able to delay the formation of cataracts, reduce peroxidation products, and improve cellular antioxidant capacity in an animal model induced by 50% galactose [29]. Because of the strong activity of Sal A, an arginine-glycine-aspartic acid-conjugated polyethyleneimine particle loaded with Sal A has been created for choroidal neovascularization-targeted antiangiogenesis therapy [18].

In the present study, we explored the therapeutic effect of Sal A on MNU-induced degeneration of photoreceptor cells. The RD model induced by MNU has good reproducibility and high specificity and is widely used in studies of the pathological mechanisms of RD and in drug screening [30, 31]. A single ip of 40 to 70 mg/kg MNU in adult rodents can produce morphological and functional changes, such as a significant reduction in photoreceptor cells and a low level or disappearance of ERG waveforms on days 3 through 7, and a stable RD model can be formed [32–34]. In this experiment, 7 days after a single administration of 60 mg/kg MNU to adult mice, retinal ERG analyses indicated a clear damage to the tissue, and the retinal ONL thickness was significantly reduced. It has been found that the apoptosis of photoreceptor cells induced by MNU is closely related to oxidative stress, and reactive oxygen species (ROS) have been considered to be a key factor in the apoptosis of photoreceptor cells [4, 35]. ROS activate members of the Bax/Bak family of proteins, and this activation ultimately leads to a caspase-mediated apoptosis cascade [3, 36]. In this study, the retinal SOD activity of mice treated with MNU decreased with time, while the level of MDA increased over time. As SOD is a key enzyme involved in scavenging-free radicals, and MDA levels are a proxy for ROS-mediated damage to lipids; these results support the idea that MNU-induced damage to retinal tissue is associated with oxidative stress.

In the present study, it was shown that Sal A did not affect the waveform of retinal ERG or retinal ONL thickness in normal mice, but it counteracted the decline of the b-wave in the ERG of mice treated with MNU, thereby improving the electrophysiology of retinas of MNU-treated mice. Sal A was also found to maintain ONL thickness in this mice model of RD. Daily administration of Sal A at 0.5 mg/kg and at 1.0 mg/kg had significant dose-dependent protective effects. These results are consistent with the conclusion that Sal A treatment can at least partially alleviate MNU-induced retinal morphological and functional damage.

Studies on the mechanism of the protective effect mediated by Sal A show that it can increase the activity of SOD in mice retinas and can reduce the levels of the lipid peroxidation product MDA, suggesting that its protective effect may be related to the enriching of endogenous antioxidants. This enrichment would relieve MNU-induced oxidative stress in retinal tissues. Through Western blotting and RT-PCR experiments, effects of MNU and Sal A on the expression of the proapoptotic genes Bax and caspase 3 and the antiapoptotic gene Bcl-2 were detected. It was found that Sal A can increase the levels of Bcl-2 mRNA and decrease the levels of Bax and caspase 3 mRNA within the retina, indicating that its protective effect is closely related to an antiapoptotic mechanism.

In addition, we studied the effects of MNU and Sal A *in vitro*. We found that the treatment of cultured 661 W cells with 1 *μ*M MNU can induce damage and reduce cell viability, which is consistent with literature reports [15]. Other *in vitro* studies have shown that Sal A can inhibit H_2_O_2_-induced reductions of retinal pigment epithelial cell viability by inhibiting apoptosis and reducing ROS production [19]. It has also been found to protect oxidized LDL-induced retinal pigment epithelial cells from inflammation and oxidative damage [37, 38]. In the present study, we showed that treatment of normally cultured 661 W cells with Sal A is not associated with observable toxic effects. Importantly, though, treatment with Sal A can protect these cells against the damage caused by MNU and can delay MNU-induced decreases of cell viability.

## 5. Conclusions

In conclusion, our study shows that Sal A can ameliorate MNU-induced photoreceptor degeneration *in vitro* and *in vivo*. Moreover, its mechanism is closely related to antioxidation and antiapoptosis. Sal A should thus be examined further as a potential safe and effective new therapy for the clinical treatment of RD.

## Figures and Tables

**Figure 1:** Chemical structure of Sal (A). Molecular formula: C_26_H_22_O_10_; M.W.:494.45.

**Figure 2:** Results of ERGs performed under scotopic and photopic conditions. (a): Representative waveforms of scotopic and photopic ERGs from mice at day 7 post-MNU treatment. (b): Quantitative analysis of scotopic and photopic ERG b-wave amplitudes (*n* = 10). ^*∗*^*P* < 0.05, ^*∗∗*^*P* < 0.01 vs. NC group; ^#^*P* < 0.05, ^##^*P* < 0.01 vs. MNU group; ^◇^*P* < 0.05, ^◇◇^*P* < 0.01 MNU + Sal A (1.0) vs. MNU + Sal A (0.5).

**Figure 3:** Changes in retinal morphology of mice in each group on day 7 after MNU treatment. (a): Representative photograph of the central retina sectioned along the vertical axis (×400). (b): Histogram analysis of ONL thickness in each group (*n* = 10). ^*∗*^*P* < 0.05, ^*∗∗*^*P* < 0.01 vs. NC group; ^#^*P* < 0.05, ^##^*P* < 0.01 vs. MNU group; ^◇^*P* < 0.05, ^◇◇^*P* < 0.01 MNU + Sal A (1.0) vs. MNU + Sal A (0.5).

**Figure 4:** Histogram analysis of SOD activity and MDA content in retina of mice in each group on day 3 (D3) and day 7 (D7) (*n* = 10). ^*∗*^*P* < 0.05, ^*∗∗*^*P* < 0.01 vs. NC group; ^#^*P* < 0.05, ^##^*P* < 0.01 vs. MNU group; ^◇^*P* < 0.05, ^◇◇^*P* < 0.01 MNU + Sal A (1.0) vs. MNU + Sal A (0.5). ^▲^*P* < 0.05, ^▲▲^*P* < 0.01 vs. the value at day 3 in the same group.

**Figure 5:** (a): Western blotting was utilized to compare Bax, caspase 3, and Bcl-2 protein expression in the retinas of mice in each group. (b): Levels of Bax, Bcl-2, and caspase 3 protein expression in each group's retinal tissues were measured (*n* = 10). ^*∗*^*P* < 0.05, ^*∗∗*^*P* < 0.01 vs. NC group; ^#^*P* < 0.05, ^##^*P* < 0.01 vs. MNU group; ^◇^*P* < 0.05, ^◇◇^*P* < 0.01 MNU + Sal A (1.0) vs. MNU + Sal A (0.5). ^▲^*P* < 0.05, ^▲▲^*P* < 0.01 vs. the value at day 3 in the same group.

**Figure 6:** Changes of mRNA in the levels of expression of Bax, caspase 3, and Bcl-2 in the retinas of mice in each group. The levels of expression of the mRNA of the three indicators on day 3 (D3) and day 7 (D7) of the treatment regimen as determined by RT-PCR. Data were normalized to the expression of the mRNA coding for *β* actin (*n* = 10). ^*∗*^*P* < 0.05, ^*∗∗*^*P* < 0.01 vs. NC group; ^#^*P* < 0.05, ^##^*P* < 0.01 vs. MNU group; ^◇^*P* < 0.05, ^◇◇^*P* < 0.01 MNU + Sal A (1.0) vs. MNU + Sal A (0.5). ^▲^*P* < 0.05, ^▲▲^*P* < 0.01 vs. the value at day 3 in the same group.

**Figure 7:** (a):Morphologies of 661 W cells at 12 and 24 h after treatment. 661 W cells in each group were observed with an inverted light microscope (×100). (b) Cell viability of 661 W cell line upon the noted treatment (*n* = 10). ^*∗*^*P* < 0.05, ^*∗∗*^*P* < 0.01 vs. NC group; ^#^*P* < 0.05, ^##^*P* < 0.01 vs. MNU group; ^◇^*P* < 0.05, ^◇◇^*P* < 0.01 vs.12 h value in the same group.

## Data Availability

No data were used to support this study.
